The article "Lung Cancer: MicroRNA and Target Database" was retracted in 2012. Reason: no approval from an author.

# Lung Cancer: MicroRNA and Target Database

**DOI:** 10.3779/j.issn.1009-3419.2012.07.07

**Published:** 2012-07-20

**Authors:** Challa KIRAN, Ponnala DEEPIKA

**Affiliations:** Centre for Cellular and Molecular Biology, India

**Keywords:** Lung neoplasms, MicroRNAs, Targets

## Abstract

MicroRNAs (miRNAs) are a class of non-coding RNAs that hybridize to mRNAs and induce either translation repression or mRNA cleavage. Recently, it has been reported that miRNAs could possibly play a critical role in cellular processes like regulation of cell growth, differentiation, and apoptosis, emphasizing their role in tumorigenesis. Likewise, several miRNA's are involved in lung cancer tumorigenesis. The present review puts forth a database of human miRNA's involved in lung cancer along with their target genes. It also provides sequences of miRNA's and their chromosomal locations retrieved from different databases like microCosm (218 microRNAs), PhenomiR (293 microRNAs), and mir2Disease (90 microRNAs) and target gene information such as the pathways like cell cycle regulation, angiogenesis, apoptosis etc. Though miRNA's are still to be explored, they hold a promise as therapeutic targets and diagnostic markers of cancer.

## Introduction

MicroRNAs (miRNA) are short, noncoding RNAs regulating gene expression^[1, 2]^. MicroRNAs were discovered in 1993 by Victor Ambros and group. However, their importance as an abundant class of regulatory non-coding RNAs came into light only after their rediscovery by Reinhart^[3]^. MicroRNAs are reported to cover 1% to 3% of the genomes and 30% of the genes are shown to be regulated by them (Lai^[4]^). Thousands of miRNAs involved in various human diseases have been identified by Jin^[5]^. The reason for their involvement is mainly due to a change in the copy numbers or due to mutations in the sequence of miRNA or their target sites^[6]^. They were also shown to be deregulated in majority of cancers^[7]^. Recent studies have demonstrated the critical role of miRNAs in cancer pathogenesis^[8-14]^. The potential of restoring levels of aberrantly under expressed miRNAs with miRNA mimics or inactivating over-expressed miRNAs with miRNA inhibitors has been explored and shows promise as the next generation of therapeutic strategies^[15-19]^.

Lung cancer is one of the most common causes of cancer related deaths in the world and is responsible for 1.3 million deaths worldwide every year. Lung cancer can be divided into two groups according to pathology: non-small cell lung cancer (NSCLC) (80.4%) and small cell lung cancer (SCLC) (16.8%)^[20]^. Many factors potentially contribute to lung cancer formation for e.g. tobacco smoke, ionizing radiations and viral infections. However, the mechanisms involved in lung carcinogenesis remain largely unknown. Lung cancer is initiated by activation of oncogenes or inactivation of tumor suppressor genes^[21]^. Similar to other cancers, many pathways are involved in lung cancer development and progression.

The article "Lung Cancer: MicroRNA and Target Database" was retracted in 2012. Reason: no approval from an author.

MicroRNAs are involved in many pathways related to lung cancer. ErbB2 (HER2/Neu), ErbB3 and ErbB4 belong to the family of receptor tyrosine kinases. These kinases initiate signal cascades leading to DNA synthesis and cell proliferation, and their over-expression is often critically involved in tumorigenesis and cancer cell proliferation^[22]^. The epidermal growth factor receptor (EGFR)/ErbB1 regulates cell proliferation, apoptosis, angiogenesis and tumor invasion in non-small cell lung carcinoma^[21]^. Recent investigations have demonstrated that miRNAs are likely to be involved in the regulation of EGFR in lung cancer. An inhibitor of miR-128b resulted in up-regulated EGFR expression in an EGFR-expressing NSCLC cell line, and treatment with a miR-128b mimic resulted in a concomitant reduction of EGFR expression^[23]^. Inhibition of miR-21 was recently shown to enhance the anti-apoptotic potential of an anti-EGFR tyrosine kinase inhibitor in an *EGFR*-mutant lung adenocarcinoma cell line^[24]^. The proto-oncogene *RAS* is the central molecule of the SOS-RAS-Raf-MAPK cascade which is the downstream cytoplasmic effector of the growth factor receptors. Approximately 20% of tumors in general and 30% of lung tumors have activating mutations in one of the *RAS* genes^[25]^. One of the downstream effectors of the RAS signaling pathway is the *MYC* oncogene. MYC amplification and over-expression have been detected in different histologic subtypes of lung cancer^[26]^. Both RAS and MYC are targets of the let-7/miR-98 family of miRNAs. Johnson ^[27]^ showed that members of the let-7 family of miRNAs bind to the 3′UTR of RAS, down-regulating RAS expression in human cells. It is seen that let-7 is poorly expressed in lung cancer compared to normal lung tissue, and that the expression of let-7 is inversely correlated with the expression of RAS in lung tumor samples^[28]^. miR-29 is down-regulated in a number of human cancers including lung cancers, and its ability to repress Mcl-1 coupled with its role in regulating epigenetic DNA methylation^[29]^ means that enhancing expression of this regulatory element could be an effective therapeutic strategy^[30-32]^. Vascular endothelial growth factor (VEGF) is an important mediator of angiogenesis during tumor development, and this molecule and its receptor (VEGFR) have been primary targets of therapies designed to target pathological angiogenic signaling^[33]^. Liu^[34]^ investigated the involvement of miR-126 in the regulation of angiogenic processes in a lung cancer model. They found decreased expression of miR-126 and increased expression of VEGF-A in various lung cancer cell lines and showed that introduction of miR-126 using a lentiviral vector could down-regulate the expression of VEGF-A and inhibit growth.

The article "Lung Cancer: MicroRNA and Target Database" was retracted in 2012. Reason: no approval from an author.

Inactivation of tumor suppressor genes plays important role in lung carcinogenesis. The *p*53 tumor suppressor gene, located on chromosome 17p, is affected in 60%-75% of lung cancer including both NSCLC and SCLC while Rb is more likely inactivated in SCLC^[35]^. In lung cancer cells, induction of miR-34 results in apoptosis^[36, 37]^ and miRNA profiling shows that the expression of miR-34a, miR-34b, and miR-34c are directly correlated with expression of the p53 tumor suppressor^[38]^, suggesting that miR-34 is involved in regulating apoptosis as a regulatory target of p53. Evidence is emerging that tumor suppressors are likely to be regulated by miRNA activity. *FUS1/TUSC2* is a tumor suppressor gene located on 3p21.3 that has been shown to be negatively regulated by the activities of miR-197, miR- 93, miR-98, and miR-378^[13, 39]^. Reduced or complete loss of Fus1 expression was found in 82% and 100% of non-small cell and small cell lung cancer cell lines^[40]^, and elevated levels of miR-93 and miR-197 have been shown to correlate with reduced Fus1 expression in NSCLC tumor specimens^[39]^. Another important tumor suppressor gene is LKB1, whose loss-of-function mutation/deletion is observed in 30% lung adenocarcinomas and 20% of squamous cell carcinomas^[41, 42]^. An investigation of miR-126 in the regulation of invasive potential in lung cancer revealed an inverse relationship between Crk and miR-126 expression in squamous cell tumors^[43]^. miR-21 also targets PDCD4, a pro-apoptotic gene that inhibits tumorigenesis and whose down-regulation has been linked to poor survival in colon and lung cancer patients^[44-46]^. The let-7 family has been shown to inhibit the expression of several oncogenes including RAS, MYC, and HMGA2^[28, 47-49]^. Several studies have implicated the miR-17-92 cluster of miRNAs as an actual oncogene with important regulatory effects on pathologic tumor cell proliferation in various tissues including breast and lung^[50-52]^.

### Lung cancer microRNAs database

All these genetic pathways play a critical role in lung cancer progression. MicroRNAs play a very important role in the regulation of these pathways. Finding the targets of miRNA is equally important as finding the miRNA itself^[53]^. Identifying these miRNAs and their target genes provides a platform to work towards the understanding of lung cancer pathogenesis. Computational prediction of target genes for miRNAs in animals is a challenging task for both experimental and computational group, due to the complexity of miRNA target recognition^[54]^.

The article "Lung Cancer: MicroRNA and Target Database" was retracted in 2012. Reason: no approval from an author.

Numerous databases are available which facilitate easy and efficient mining of microRNAs and their target genes involved in a specific cancer. Databases based on sequence annotation and microRNA genomics are miRBase^[55]^, human microRNA disease database^[56]^, miRNAMap^[57]^, and miRGen^[58]^. miRBase serves as a central database for experimentally supported mature miRNA sequences for each supported miRNA. It also provides the genomic coordinates of the predicted precursor sequences. TargetScan^[59]^, PicTar^[60]^, TargetMiner^[61]^, miRDB are the databases for miRNA target prediction and functional annotations in animals^[62]^. microRNA.org target and expression 2005, are the databases used for microRNA target predictions based on the complementary perfect base-pairing in the seed region of the targets. TarBase^[63]^ is a resource of experimentally validated microRNA targets.

However, no database exists which provides a complete overview of microRNAs controlling lung cancer pathogenesis and progression. This review puts forth a database including almost all the microRNAs involved in lung carcinogenesis. The miRNAs involved in lung cancer are pooled up from databases, MicroCosm (218 microRNAs), PhenomiR (293 microRNAs) and mir2Disease (90 microRNAs). A supplementary excel document is provided with this review which gives a detailed description of the MiRNA's involved in lung cancer. It also includes information about the accession numbers, chromosomal positions and validated targets of the respective microRNA's.

MicroRNAs involved in lung cancer were derived from miRBase, PhenomiR^[64]^, MiR2Disease database^[56]^. After manually curating the miRNAs from different databases accession numbers and sequences of microRNAs were collected from the miRBase database. MicroRNAs chromosome positions were obtained from the *HUGO* gene nomenclature committee (HGNC). PhenomiR database contains the microRNA expression levels in the different lung cancer samples and cell lines, those were collected for specific microRNAs which are present in PhenomiR database and related to lung cancer.

### Experimentally validated target interactions

Experimentally validated targets for these lung cancer microRNAs were collected from the mir2disease and TarBase databases. These target genes were submitted to gene Go analysis software. Gene Go is the pathway analysis software which gives the information about interaction between the different biological molecules. Many target genes were found to be involved in lung cancer development and progression and these proteins are present in extracellular, membrane, cytoplasm and nucleus. All these target genes are positively or negatively regulated by the each other. Receptor ligand, generic kinase, transcription factors, lipid phosphatase, generic phosphatase, generic binding proteins and RAS super family proteins have been found to be involved in the lung cancer development. Generic binding proteins like cyclin D1, P27KIP1, and BCL2 are very important molecules in the cytoplasmic region and regulate many other targets. C-Myc is one of the important transcription factor which is present in the nucleus and regulates many proteins in the cytoplasmic region. Interactions between the extracellular, membranes, cytoplasmic and nuclear proteins are shown in the Fig 1.

**1:** Lung cancer target interactions between the extracellular, membranes, cytoplasmic and nuclear proteins

The major pathways associated in lung cancer based on genego analysis are pathways involving cell proliferation, cell cycle regulation, angiogenesis, signal transduction and apoptosis. The significant protein found to regulate most of the other proteins is c-Myc and the proteins regulated by c-Myc are cyclins, cyclin dependant kinases (CDKs), DNA methyl transferases, and CDK inhibitors. C-Myc is a basic-helix-loop-helix/leucine zipper (bHLH/LZ) transcription factor that controls the G_1_-S cell-cycle transition and is over expressed in many human tumors. A thorough analysis of the pathway circuit produced by genego software depicts that C-myc directly or indirectly regulates most of the proteins which involve in various other pathways. Thus c-Myc is a potent protein which needs to be studied.

The article "Lung Cancer: MicroRNA and Target Database" was retracted in 2012. Reason: no approval from an author.

It is also seen that p27KIP1 too regulates quite a few proteins. p27KIP1 is a cell-cycle regulatory protein that interacts with cyclin-CDK2 and -CDK4, inhibiting cell cycle progression at G_1_. But an altered expression of p27KIP1 dysregulates the expression of proteins involved in cell cycle regulation and thereby leads to cell proliferation. Interestingly, the pathway circuit obtained from genego software reveals that c-Myc indirectly regulates p27KIP1 through Bcl2 and H-Ras. Hence c-Myc becomes further more a vital protein to be focused on, apart from p27KIP1.

MicroRNA regulation of lung cancer-related pathways provides numerous opportunities for therapeutic intervention. Competitive inhibition of miRNAs or the delivery of exogenously produced miRNAs could provide substantial therapeutic benefit by reducing the activity of prooncogenic miRNAs. These approaches are still in the preclinical stages, although intriguing evidence is emerging that supports their use in clinical applications. Expression of miR-29 family members has been shown to reduce tumorigenic potential in a lung cancer model^[29]^. Exogenous delivery of a synthetic let-7 mimic has been used to mediate remission of established NSCLC tumors in mice^[28]^. Future work will focus on both chemical modifications and delivery vehicles in order to maximize the therapeutic benefits and minimize the side effects of strategies designed to alter intracellular levels of specific miRNAs (Fig 2).

**2:** Venn diagram showing the distribution of total microRNAs identified form different databases. The numbers indicate the total microRNAs identified from each category and the number of microRNAs commonly identified between them.

## Conclusion

The study of microRNAs has evolved rapidly since the discovery of this important class of regulatory molecules. The proposed lung cancer microRNA database would prove to be helpful to lung cancer biologists in one or the other way. Further studies on the miRNA's listed in the database would explore and explain the relation between miRNAs and the initiation and progression of malignant neoplasias and the basic biological roles that they play in tumor cell survival, invasion, metastasis, and angiogenesis. However, many issues are still to be addressed before the miRNAs can be used as therapeutic tools in the field of oncology. miRNA dysregulation in particular tumor subtypes need to be further investigated, which may aid the development of new therapies that specifically target tumor cells with particular molecular and regulatory profiles. Overall, miRNAs are ubiquitous regulatory molecules that hold great promise for increasing our understanding of lung cancer and for improving upon current diagnostic and therapeutic methods. Further evaluation of their value in cancer diagnostics and of the functional consequences of their manipulation will provide researchers and oncologists with a wealth of new tools to characterize and treat this prevalent and diverse disease.

## References

[1] Ambros V (2004). The functions of animal microRNAs. Nature.

[2] Garzon R, Fabbri M, Cimmino A (2006). MicroRNA expression and function in cancer. Trends Mol Med.

[3] Reinhart BJ, Weinstein EG, Rhoades MW (2002). MicroRNAs in plants. Genes & Dev.

[4] Lai EC, Tomancak P, Williams RW (2003). Computational identification of Drosophila microRNA genes. Genome Biol.

[5] Jin P, Zarnescu DC, Ceman S (2004). Biochemical and genetic interaction between the fragile X mental retardation protein and the microRNA pathway. Nat Neurosci.

The article "Lung Cancer: MicroRNA and Target Database" was retracted in 2012. Reason: no approval from an author.

[6] Meola N, Gennarino VA, Banfi S (2009). MicroRNAs and genetic diseases. Pathogenetics.

[7] Calin GA, Liu CG, Sevignani C (2004). MicroRNA profiling reveals distinct signatures in B cell chronic lymphocytic leukemias. Proc Natl Acad Sci USA.

[8] He L, He X, Lowe SW (2007). MicroRNAs join the p53 network-Another piece in the tumour-suppression puzzle. Nat Rev Cancar.

[9] Cho WC (2007). OncomiRs: The discovery and progress of microRNAs in cancers. Mol Cancer.

[10] Hwang HW, Mendell JT (2006). MicroRNAs in cell proliferation, cell death, and tumorigenesis. Br J Cancer.

[11] Esquela-Kerscher A, Slack FJ (2006). J Oncomirs-microRNAs with a role in cancer. Nat Rev Cancer.

[12] Hebert C, Norris K, Scheper MA (2007). High mobility group A2 is a target for miRNA-98 in head and neck squamous cell carcinoma. Mol Cancer.

[13] Lee DY, Deng Z, Wang CH (2007). MicroRNA-378 promotes cell survival, tumor growth, and angiogenesis by targeting SuFu and Fus-1 expression. Proc Natl Acad Sci USA.

[14] O'Donnell KA, Wentzel EA, Zeller KI (2005). c-Myc-regulated microRNAs modulate E2F1 expression. Nature.

[15] Mercatelli N, Coppola V, Bonci D (2008). The inhibition of the highly expressed miR-221 and miR-222 impairs the growth of prostate carcinoma xenografts in mice. PLoS One.

[16] Felicetti F, Errico MC, Bottero L (2008). The promyelocytic leukemia zinc finger-microRNA-221/-222 pathway controls melanoma progression through multiple oncogenic mechanisms. Cancer Res.

[17] Wickramasinghe NS, Manavalan TT, Dougherty SM (2009). Estradiol downregulates miR-21 expression and increases miR-21 target gene expression in MCF-7 breast cancer cells. Nucleic Acids Res.

[18] Yang Y, Chaerkady R, Beer MA (2009). Identification of miR-21 targets in breast cancer cells using a quantitative proteomic approach. Proteomics.

[19] Si ML, Zhu S, Wu H (2007). miR-21-mediated tumor growth. Oncogene.

[20] Jemal A, Siegel R, Ward E (2008). Cancer statistics, 2008. CA Cancer J Clin.

[21] Herbst RS, Heymach JV, Lippman SM (2008). Lung cancer. N Engl J Med.

[22] Holbro T, Beerli RR, Maurer F (2003). The ErbB2/ErbB3 heterodimer functions as an oncogenic unit: ErbB2 requires ErbB3 to drive breast tumor cell proliferation. Proc Natl Acad Sci USA, the United States of America.

[23] Weiss GJ, Bemis LT, Nakajima E (2008). EGFR regulation by microRNA in lung cancer: Correlation with clinical response and survival to gefitinib and EGFR expression in cell lines. Ann Oncol.

[24] Seike M, Goto A, Okano T (2009). MiR-21 is an EGFR-regulated antiapoptotic factor in lung cancer in never-smokers. Proc Natl Acad Sci USA.

[25] Bos JL (1989). Ras oncogenes in human cancer: A review. Cancer Res.

The article "Lung Cancer: MicroRNA and Target Database" was retracted in 2012. Reason: no approval from an author.

[26] Zajac-Kaye M (2001). Myc oncogene: A key component in cell cycle regulation and its implication for lung cancer. Lung Cancer.

[27] Johnson SM, Grosshans H, Shingara J (2005). RAS is regulated by the let-7 microRNA family. Cell.

[28] Kumar MS, Erkeland SJ, Pester RE (2008). Suppression of non-small cell lung tumor development by the let-7 microRNA family. Proc Natl Acad Sci USA.

[29] Fabbri M, Garzon R, Cimmino A (2007). MicroRNA-29 family reverts aberrant methylation in lung cancer by targeting DNA methyltransferases 3A and 3B. Proc Natl Acad Sci USA.

[30] Yanaihara N, Caplen N, Bowman E (2006). Unique microRNA molecular profiles in lung cancer diagnosis and prognosis. Cancer Cell.

[31] Calin GA, Ferracin M, Cimmino A (2005). A microRNA signature associated with prognosis and progression in chronic lymphocytic leukemia. N Eng J Med.

[32] Cummins JM, He Y, Leary RJ (2006). The colorectal microRNAome. Proc Natl Acad Sci USA.

[33] Kerbel RS (2008). Tumor angiogenesis. N England J Med.

[34] Liu B, Peng XC, Zheng XL (2009). MiR-126 restoration down-regulate VEGF and inhibit the growth of lung cancer cell lines *in vitro* and *in vivo*. Lung Cancer.

[35] Devereux TR, Taylor JA, Barrett JC (1996). Molecular mechanisms of lung cancer. Interaction of environmental and genetic factors. Giles F. Filley Lecture. Chest.

[36] Tarasov V, Jung P, Verdoodt B (2007). Differential regulation of microRNAs by p53 revealed by massively parallel sequencing: miR-34a is a p53 target that induces apoptosis and G_1_-arrest. Cell Cycle.

[37] Hermeking H (2010). The miR-34 family in cancer and apoptosis. Cell Death Differ.

[38] He L, He X, Lim LP (2007). A microRNA component of the p53 tumour suppressor network. Nature.

[39] Du L, Schageman JJ, Subauste MC (2009). miR-93, miR-98, and miR-197regulate expression of tumor suppressor gene *FUS1*. Mol Cancer Res.

[40] Prudkin L, Behrens C, Liu DD (2008). Loss and reduction of FUS1 protein expression is a frequent phenomenon in the pathogenesis of lung cancer. Clin Cancer Res.

[41] Ji H, Ramsey MR, Hayes DN (2007). LKB1 modulates lung cancer differentiation and metastasis. Nature.

[42] Ding L, Getz G, Wheeler DA (2008). Somatic mutations affect key pathways in lung adenocarcinoma. Nature.

[43] Crawford M, Brawner E, Batte K (2008). MicroRNA-126 inhibits invasion in non-small cell lung carcinoma cell lines. Biochem Biophys Res Commun.

[44] Jansen AP, Camalier CE, Colburn NH (2005). Epidermal expression of the translation inhibitor programmed cell death 4 suppresses tumorigenesis. Cancer Res.

[45] Chen Y, Knösel T, Kristiansen G (2003). Loss of PDCD4 expression in human lung cancer correlates with tumour progression and prognosis. J Pathol.

The article "Lung Cancer: MicroRNA and Target Database" was retracted in 2012. Reason: no approval from an author.

[46] Mudduluru G, Medved F, Grobholz R (2007). Loss of programmed cell death 4 expression marks adenoma-carcinoma transition, correlates inversely with phosphorylated protein kinase B, and is an independent prognostic factor in resected colorectal cancer. Cancer.

[47] Sampson VB, Rong NH, Han J (2007). MicroRNA let-7a down-regulates MYC and reverts MYC-induced growth in Burkitt lymphoma cells. Cancer Res.

[48] Mayr C, Hemann MT, Bartel DP (2007). Disrupting the pairing between let-7 and Hmga2 enhances oncogenic transformation. Science.

[49] Lee YS, Dutta A (2007). The tumor suppressor microRNA let-7 represses the *HMGA2* oncogene. Genes Dev.

[50] Hayashita Y, Osada H, Tatematsu Y (2005). A polycistronic microRNA cluster, miR-17-92, is overexpressed in human lung cancers and enhances cell proliferation. Cancer Res.

[51] He L, Thomson JM, Hemann MT (2005). A microRNA polycistron as a potential human oncogene. Nature.

[52] Mendell JT (2008). miRiad roles for the miR-17-92 cluster in development and disease. Cell.

[53] Bartel DP (2004). MicroRNAs: genomics, review biogenesis, mechanism, and function. Cell,.

[54] Enright AJ, John B, Gaul U (2003). MicroRNA targets in Drosophila. Genome Biol.

[55] Griffiths-Jones S, Saini HK, van Dongen S (2008). miRBase: tools for microRNA genomics. Nucleic Acids Res.

[56] Jiang Q, Wang Y, Hao Y (2009). miR2Disease: a manually curated database for microRNA deregulation in human disease. Nucleic Acids Res.

[57] Hsu PW, Huang HD, Hsu SD (2006). miRNAMap: genomic maps of microRNA genes and their target genes in mammalian genomes. Nucleic Acids Res.

[58] Megraw M, Sethupathy P, Corda B (2007). miRGen: a database for the study of animal microRNA genomic organization and function. Nucleic Acids Res.

[59] Lewis BP, Shih IH, Jones-Rhoades MW (2003). Prediction of mammalian microRNA targets. Cell.

[60] Krek A, Grün D, Poy MN (2005). Combinatorial microRNA target predictions. Nat Genet.

[61] Bandyopadhyay S, Mitra R (2009). TargetMiner: microRNA target prediction with systematic identification of tissue-specific negative examples. Bioinformatics.

[62] Wang X (2009). A PCR-based platform for microRNA expression profiling studies. RNA.

[63] Sethupathy P, Megraw M, Hatzigeorgiou AG (2006). A guide through present computational approaches for the identification of mammalian microRNA targets. Nat Methods.

[64] Ruepp A, Kowarsch A, Schmidl D (2010). PhenomiR: a knowledgebase for microRNA expression in diseases and biological processes. Genome Biology.

